The article "Influenza A virus infection engenders a poor antibody response against the ectodomain of matrix protein 2" was published in 2006. Journal: Virol J.

# Influenza A virus infection engenders a poor antibody response against the ectodomain of matrix protein 2

**DOI:** 10.1186/1743-422X-3-102

**Published:** 2006-12-06

**Authors:** JingQi Feng, Manxin Zhang, Krystyna Mozdzanowska, Darya Zharikova, Henry Hoff, William Wunner, Robert B Couch, Walter Gerhard

**Affiliations:** 1 Immunology Program, The Wistar Institute, 3601 Spruce Street, Philadelphia PA 19104-4268, USA; 2 Baylor College of Medicine, Houston, TX 77030-3498, USA

## Abstract

**Background:**

Matrix protein 2 (M2) is an integral tetrameric membrane protein of influenza A virus (IAV). Its ectodomain (M2e) shows remarkably little diversity amongst human IAV strains. As M2e-specific antibodies (Abs) have been shown to reduce the severity of infection in animals, M2e is being studied for its capability of providing protection against a broad range of IAV strains. Presently, there is little information about the concentration of M2e-specific Abs in humans. Two previous studies made use of ELISA and Western blot against M2e peptides and recombinant M2 protein as immunosorbents, respectively, and reported Ab titers to be low or undetectable. An important caveat is that these assays may not have detected all Abs capable of binding to native tetrameric M2e. Therefore, we developed an assay likely to detect all M2e tetramer-specific Abs.

**Results:**

We generated a HeLa cell line that expressed full length tetrameric M2 (HeLa-M2) or empty vector (HeLa-C10) under the control of the tetracycline response element. These cell lines were then used in parallel as immunosorbents in ELISA. The assay was standardized and M2e-specific Ab titers quantified by means of purified murine or chimeric (mouse variable regions, human constant regions) M2e-specific Abs in the analysis of mouse and human sera, respectively. We found that the cell-based ELISA was substantially more effective than immobilized M2e peptide in detecting M2e-specific Abs in sera of mice that had recovered from repetitive IAV infections. Still, titers remained low (< 5 μg/ml) even after two consecutive infections but increased to ~50 μg/ml after the third infection. Competition with free M2e peptide indicated that ~20% of M2e-specific Abs engendered by infection reacted with M2e peptide. In humans presenting with naturally acquired influenza virus infection, 11 of 24 paired sera showed a ≥ 4-fold increase in M2e-specific Ab titer. The Ab response appeared to be of short duration as titers were very low (average 0.2 μg/ml) in all patients at onset of infection and in controls, in spite of evidence for previous exposure to IAV.

**Conclusion:**

The results provide convincing evidence that M2e-specific Ab-mediated protection is currently lacking or suboptimal in humans.

## Background

Matrix protein 2 (M2) is a 97 aa-long transmembrane protein of IAV [1]. It contains a 24 aa-long (23 aa after posttranslational removal of the N-terminal Met) non-glycosylated N-terminal ectodomain (M2e). The mature protein forms homotetramers [2,3] that are displayed at high density (~50% of density of hemagglutinin (HA) trimers) in the plasma membrane of infected cells during the stage of virus maturation [1,4] but at low density (1–2% of HA) in the membrane of mature virus particles [5]. The protein exhibits pH-inducible proton transport activity and regulates the pH of the viral core during virus entry into the host cell and of transport vesicles that deliver viral transmembrane proteins to the plasma membrane for virus assembly [6,7].

There has been growing interest in M2 as a "universal" vaccine that may protect against a much wider range of IAVs than current vaccines. The potential of M2 as "universal" vaccine derives from the following observations: First, antibodies (Abs) directed against its ectodomain (M2e) have been shown to restrict virus replication and reduce severity of disease in animal models [4,8-18], though they are less protective than HA-specific Abs and cannot provide "sterilizing immunity" or clear an infection on their own [4]. Second, M2e shows a remarkably high degree of structural conservation amongst human IAV strains. This is demonstrated in Fig 1, which shows the M2e aa composition of 1505 IAVs isolated from humans between 1918 and 2005. Third, humans currently appear to lack M2e-specific Ab-mediated protection. This has been indicated by two studies that measured M2 specific Ab titers in human sera. In one of these [19], paired serum samples from the acute and convalescent phase of 17 patients presenting with naturally acquired influenza virus infection were tested by ELISA and Western blot for Abs reactive with full-length M2 generated in the baculovirus system. By ELISA, 5 (35%) convalescent sera showed a rise of ≥ 2-fold in M2-specific and 15 (88%) in nucleoprotein (NP)-specific Ab titer [19]. The Western blot appeared to be more sensitive as it detected M2-specific Abs in 13 (70%) convalescent serum samples. Importantly, however, no M2-specific Abs could be detected in acute serum samples, which was in marked contrast to NP-specific Abs, which were detectable by ELISA and apparently resulted from previous infections or vaccinations (NP is a relatively conserved IAV protein). Similarly, no significant differences in Ab titers could be detected between sera from 66 patients with influenza and 44 influenza negative individuals when tested by ELISA against M2e peptide immunosorbent [20]. Taken together, these studies indicated that M2-specific Ab responses were inconsistently and poorly induced in humans by IAV infection and, if induced, appeared to be of low titer and short duration. Similar findings were made in mice, in which recovery from pulmonary infection also did not result in substantial M2e-specific Ab titers when measured by ELISA against M2e peptide [10,11,13].

**Figure 1:** **M2e sequence diversity amongst human influenza A virus isolates**. The sequence of 1505 human isolates (records in public data banks on August 17, 2006) of H1N1, H1N2, H2N2, H3N2, H5N1 and H9N2 subtypes is represented as a percentage of the M2e consensus sequence, which is listed in single amino acid code on the left from top to bottom, excluding the postranslationally removed methionine. Observed replacement mutations are listed on the right side by single amino acid code and their overall frequency is indicated by the gray portions of the horizontal bars.

An important caveat with regard to the low/absent M2e-specific Ab responses is the possibility that previously used assays failed to detect the entire repertoire of M2e-specific Abs. The main M2 immunogen generated in the course of infection is presumably the native M2 homotetramer, but only a fraction of native tetramer-specific Abs may react with denatured M2 protein in Western blot [19] or monomeric M2e peptides coated onto plastic [20]. To avoid this shortcoming, we previously used virus-infected MDCK cells as immunosorbents to measure the M2e-specific Ab response in mice immunized with M2e-specific vaccines [13]. However, because virus-infected cells express a variety of IAV proteins, this assay could not be used to measure M2e-specific Abs in sera from hosts that have been exposed to IAV. Therefore, we generated an adherent HeLa cell line that stably expressed full-length tetrameric M2 under the control of the tetracycline response element (Tet) and used it as an immunosorbent in ELISA. We found that HeLa-M2 immunosorbents detected higher Ab titers than M2e-peptide immunosorbents in sera of mice immunized by IAV infection. The results indicated that ~80% of the M2e-specific Abs engendered by infection reacted exclusively with cell-expressed (tetrameric) M2e. Still, M2e-specific Ab titers remained low (< 5 μg/ml), even after two consecutive infections, while NP-specific titers reached maximum levels (50–100 μg/ml) after the first infection. Measurement of M2e-specific Ab titers in paired serum samples from the acute and convalescent phase of humans presenting with natural IAV infection revealed a very low M2e-specific Ab titer (average 0.2 μg/ml) in acute serum samples and a ≥ 4-fold increase in only 50% of the patients. Taken together, the results confirmed the generally poor induction of the M2e-specific Ab response by IAV infection and indicated that humans currently lack optimal M2e-specific protection. This provides an important reason for development of an M2e-specific vaccine.

## Results

### Development of the HeLa-M2 ELISA

M2-specific Ab responses have been measured previously by assays that used extracts of cells infected with M2-recombinant baculovirus [19] or M2e-peptides and peptide conjugates as immunosorbents [10,13,14,20]. These immunosorbents may not detect the entire repertoire of Abs capable of reacting with native tetrameric M2e displayed in the plasma membrane of infected host cells. We therefore decided to develop an ELISA that used an M2-transfected adherent cell line as immunosorbent. Transfection of various types of target cells with an expression vector encoding the full-length PR8-M2-GFP fusion protein resulted in good transient expression but generation of a stable transfected cell line consistently failed (data not shown). We suspected that this failure may be the consequence of an inhibitory effect of M2 expression on cell metabolism or growth, as has been suggested by other investigators [21]. Culture of transfected cells in the presence of the M2 inhibitor amantadine did not improve selection of stable transfectants, which is in agreement with the fact that PR8 is resistant to this inhibitor [5]. We then turned to the "Tet-on" expression system, in which M2 is under the control of the minimal CMV promoter and tetracycline response element. In this system, the constitutive expression of the inserted transgene is minimal but can be increased by addition of tetracycline or doxycycline to the culture medium. Stable M2-transfectants could be selected in this controlled expression system. Although the selected HeLa-M2 line turned out to be quite leaky for M2 expression in the absence of doxycycline (Figure 2A), it could nevertheless be propagated in long-term culture and M2 expression could be further enhanced by treatment of the cells for two days with doxycycline (1 μg/ml) prior to their use as immunosorbents in ELISA (Figure 2A). To control for non-specific Ab binding in the ELISA, we also generated a HeLa cell line (HeLa-C10) that was stably transfected with empty vector.

**Figure 2:** **Antigenicity of HeLa-M2 cells**. A. HeLa-M2 cell immunosorbents were prepared in medium without (diamonds) or with (circles) doxycycline (1 μg/ml) and tested for reaction with the M2e-specific MAb 14C2-S1-4 (filled symbols) or HA-specific MAb H36-4-5.2 (open symbols). Bound MAb was detected by ELISA as described in the Method section. Symbols indicate mean OD_(490–750) _of triplicates. B. HeLa-M2 immunosorbent plates were prepared as described in the Method section. Plates, stored for different lengths of time in the refrigerator, were tested in ELISA with M2e-specific MAb 14C2-S1-4. Three independent assays, each indicated with a distinct symbol, were performed with distinct sets of HeLa-M2 plates that differed in storage time. In each assay, the saturation binding (OD) of the MAb was determined and expressed as a percentage of the plate with the highest saturation binding (defined as 100%) seen in the given assay. Linear regression analysis of the data indicated a relation of y = -0.46x +100 between antigenic activity (y) and days of storage (x) at 4–7°C.

Cellular immunosorbents were prepared in flat bottom 96-well polystyrene plates as described in the Method section. The cells were cultured for 2 days in the presence of doxycycline and then fixed for 20 min with 0.05% glutaraldehyde and stored in the refrigerator with PBSN-1% BSA medium until used for assay. The plates could be stored for several weeks without major loss of antigenic activity (Figure 2B). Glutaraldehyde-fixed HeLa cells exhibited a high endogenous alkaline phosphatase activity that could not be inhibited by levamisol (data not shown) but a low endogenous peroxidase activity. This made the use of a peroxidase-based ELISA system highly preferable.

As judged by ELISA against HeLa-C10 immunosorbent, sera showed substantial and individually distinct background binding in the HeLa ELISA. Therefore, each serum was routinely tested in parallel on HeLa-M2 and HeLa-C10 immunosorbents, which were both present on the same assay plate (Fig 3A–C). M2-specific binding activity was then computed as the difference in OD (Δ OD) between HeLa-M2 and HeLa-C10 immunosorbents and used to estimate the M2e-specific Ab concentration by comparison to the titration curve generated with purified M2e-specific MAb 14C2-S1-4. The suitability of this method for quantification of M2e-specific Ab titers was tested with artificial mixtures of MAb 14C2-S1-4 and naive mouse serum (NMS). As shown in Fig 3, specific binding was increasingly suppressed by increasing serum concentration. Nevertheless, 0.1 μg of MAb in 20% NMS (corresponding to 0.5 μg MAb/ml neat serum) could be reasonably well quantified as long as the quantification was based only on ΔODs seen at the trailing edge of the titration curve (Fig 3C). Because of this inhibitory effect, sera were tested at concentrations of ≤ 1/10. Given an assay-sensitivity of ~10 ng/ml, the threshold of M2e-specific Ab detection in sera was ~0.1 μg/ml.

**Figure 3:** **Effect of serum concentration on the HeLa-M2 ELISA**. Preparations of MAb 14C2-S1-4 at 0.1 μg/ml in diluents containing various concentrations (0, 5, 10, 20%, A-D) of NMS were tested in ELISA for binding to HeLa-M2 (filled circle) and HeLa-C10 (open circle). The difference in OD (Δ OD) between HeLa-M2 and HeLa-C10 is plotted in red. Δ OD was subsequently used to estimate the concentration of M2e-specific Ab in serum-containing preparations. The symbols show means of triplicates ± SEM. A representative example of several independent experiments is shown, in which different NMS samples and MAb concentrations were tested.

To determine whether M2 was expressed in HeLa cells as tetramers, cell monolayers were fixed for 20 min with glutaraldehyde (bivalent cross-linking fixative) or left unfixed. The cells were then solubilized, the extracts subjected to SDS PAGE under non-reducing conditions, blotted onto a PVDF membrane and analyzed with M2e-specific MAb (Fig 4A). Without fixation, the main molecular species detected in extracts of HeLa-M2 cells were monomeric (~13 kDa), dimeric (~24 kDa), and a faint band of tetrameric (~45 kDa) M2. The tetrameric species was more prominent in extracts of glutaraldehyde-fixed cells, which additionally showed a band corresponding to a trimer (~36 kDa). These findings are consistent with observations made by other investigators [2,3] and indicated that HeLa-M2 cells expressed M2 in tetrameric form. As expected, no M2-specific bands were detected in extracts of HeLa-C10 cells. Judging from the titration curves generated with M2e-specific MAbs (Fig 4B) and sera from M2e-MAP-immunized mice (Fig 4C), doxycyline-induced HeLa-M2 cells expressed more M2 than MDCK cells 8–11 hrs after infection with ~10 TCID_50 _of IAV/cell and were more effective in detecting M2e-specific Abs than infected MDCK cells.

**Figure 4:** **Form and density of M2 expression relative to PR8-infected MDCK cells**. A. Doxycycline-induced HeLa-M2 and HeLa-C10 cells, without (No) or with (Yes) prior glutaraldehyde fixation, were solubilized. Cell extracts were electrophoresed under non-reducing conditions, blotted onto a PVDF membrane and tested for presence of M2 by staining with MAb 14C2-S1-4. MW shows the position of molecular weight markers. B. M2e-specific MAbs 14C2-S1-4 (squares) and M2-1 (triangles) were tested by ELISA for binding to HeLa-M2 (filled symbols), virus-infected MDCK cells (open symbols), nine hrs after infection with 10 TCID_50 _of PR8 per cell, and the corresponding control cell immunosorbents. Symbols show mean ± SEM of triplicate Δ ODs. A representative assay of several independent repeat experiments is shown. C. Sera from mice immunized with M2e-MAP were tested as in B for binding to HeLa-M2 (filled symbols) and PR8-infected MDCK cells (open symbols). Pooled sera from two different groups of mice (square, triangle) are shown. A representative assay of several independent experiments is shown.

Taken together, the results showed that HeLa-M2 cells expressed tetrameric M2 and, following glutaraldehyde fixation, formed sensitive immunosorbents that were quite stable over several weeks of storage at 4°C.

### HeLa-M2 cells are more effective than M2e peptide immunosorbents in detecting M2e-specific Abs in sera of infection-immunized mice

Because most previous studies used peptide immunosorbents for measurement of M2e-specific Ab titers, we were interested in comparing peptide and HeLa-M2 immunosorbents for efficacy of M2e-specific Ab detection. To this end, MAbs and serum pools from mice immunized by infection or injection of M2e-MAP (M2e multiple antigenic peptide) [13] were tested in parallel for binding to HeLa-M2 and M2e-peptide immunosorbents. The latter had been prepared by coating wells of flat bottom polystyrene plates (same as used for preparation of HeLa-M2 immunodsorbents) with M2e-MAP at various concentrations. OD values increased with increasing concentration of coating peptide. The most informative results were obtained at the coating concentration of 0.2 μg/ml and are shown in Fig 5. At this coating concentration, all M2e-specific MAbs, except M2-1, reacted better with M2e peptide than with HeLa-M2 cells (Fig 5A). Similarly, sera from mice immunized with (4)M2e-MAP [13] reacted better with M2e peptide than with HeLa-M2 (Fig 5B). By contrast, sera from mice immunized by consecutive infections bound much better to HeLa-M2 than to M2e-MAP (Fig 5C). Thus, M2e-specific MAbs and Abs induced by immunization with M2e-MAP differed in fine specificity and/or avidity from those induced by infection.

**Figure 5:** **Comparison between HeLa-M2 and M2e-peptide immunosorbents**. A. Binding of MAbs to HeLa-M2 (filled symbols) and M2e-peptide immunosorbent (open symbols), formed by coating wells with 50 μl of M2e-MAP at 0.2 μg/ml. Two MAbs that exemplify the opposite extremes in binding activity of currently available M2e-specific MAbs, are shown: 14C2-S1-4 (squares) and M2-1(triangles). Each symbol shows mean OD ± SEM of triplicates. B. M2-specific binding (Δ OD) against HeLa-M2 (closed symbols) and M2e-MAP (open symbols) of two representative sera (triangle, square) from groups of mice immunized by three inoculations with (4)M2e-MAP. C. As in B, except for using sera from mice that had been immunized by three consecutive pulmonary influenza virus infections. All assays were performed at least twice and a representative assay is shown.

A possible explanation for the stronger reaction of sera from infection-immunized mice with HeLa-M2 than M2e peptide immunosorbents was that infection induced Abs to the intracytoplasmic region of M2 (in addition to M2e) and the former Abs may be detected by HeLa-M2 immunosorbents even though the cells had not been permeabilized intentionally. This possibility was tested with an antiserum specific for the C-terminus of M2. As shown in Fig 6A, this antiserum reacted with intentionally permeabilized but not with the standard HeLa-M2 immunosorbent, while M2e-specific MAbs, as expected, reacted equally well with both. Thus, without permeabilization, the HeLa-M2 ELISA appeared to detect exclusively M2e-specific Abs. This conclusion was confirmed by showing that sera from infection-immunized mice failed to react with HeLa-M2 immunosorbents that had been treated with trypsin to remove a major portion of M2e and thereby destroyed its antigenicity (Fig 6B).

**Figure 6:** **Only M2e is accessible to Ab on fixed non-permeabilized HeLa-M2 cells**. A. Control naive mouse serum (NMS), a mouse serum specific for the intracytoplasmic C terminus of M2 and M2e-specific MAb were tested for reaction with fixed HeLa-M2 and HeLa-C10 cells with (filled bars) and without (open bars) permeabilization. Mean Δ ODs of duplicates are shown. B. Fixed HeLa-M2 and HeLa-C10 immunosorbents were treated with increasing concentrations of trypsin (dilution of 2.5% is indicated) and then tested for reaction with a constant dose of M2e-specific MAb (triangles) or pooled serum from infection-immunized mice (squares). Symbols show Δ ODs (mean ± SEM of triplicates). One of two independent assays is shown.

Taken together, the results suggested that sera from infection-immunized mice contained M2e-specific Abs directed against conformational determinants displayed by tetrameric M2e but not monomeric M2e peptide. To confirm this proposition, sera and MAbs were tested for binding to HeLa-M2 in the presence of competing M2e peptide. As shown in Fig 7, the binding of M2e-specific MAbs and serum from M2e-MAP-immunized mice to HeLa-M2 was completely inhibited by M2e(2–24) peptide. By contrast, serum from infection-immunized mice was only partially inhibited. The results indicated that ~20% of the M2e-specific Abs induced by infection (pooled serum from four mice) recognized determinants shared by M2e peptide and HeLa-M2 and ~80% recognized determinants unique to HeLa-M2. The latter most likely are conformational determinants of M2e-tetramers.

**Figure 7:** **Competition of Ab binding to HeLa-M2 by free M2e peptide**. Increasing concentrations of M2e(2–24) peptide were tested for ability to inhibit the binding of a constant dose of MAbs 14C2-S1-4 (triangles pointing up) and M2-1 (triangles pointing down) or pooled sera from mice immunized by three consecutive infections (squares) or three injections of (4)M2e-MAP (circles). MAbs were tested at 1 μg/ml and sera at 1/200 dilution. Ab binding in the presence of competing M2e peptide was expressed as percent of its binding (Δ OD) in the absence of competing peptide. The results show the composite of three independent assays, each performed in triplicate. Each symbol shows the mean ± SEM of nine replicates.

### Analysis of M2e- and NP-specific Ab responses engendered in mice by infection

Sera from mice (2–5 mice/group) that had recovered from one, two or three consecutive IAV infections were tested in the HeLa-M2 ELISA. The results (Fig 8A) revealed low M2e Ab titers three weeks after primary infection (GMT = 1.9 μg/ml, n = 4 groups). The titers increased slightly, though not significantly, after recovery from a second infection by a heterosubtypic IAV (GMT = 3.0 μg/ml, n = 7 groups) and then rose significantly to 49 μg/ml (n = 2 groups of two mice each) after the third infection. The same sera were also tested for Abs directed to NP, a viral protein that is highly conserved between IAV strains. In this case (Fig 8B), close to maximum NP-specific Ab titers (GMT = 43 μg/ml, n = 5 groups) were reached after recovery from the first infection and the titers increased only slightly after a second (GMT = 51 μg/ml) and third (GMT = 60 μg/ml) infection. Thus, in spite of the improved assay, which probably is capable of detecting all biologically relevant M2e-specific Abs, the results indicated that infection engendered a poor M2e-specific Ab response in mice and that several consecutive infections were required to raise the response to the level attained by NP-specific Abs after a single infection.

**Figure 8:** **M2e- and NP-specific Ab responses of BALB/c mice convalescent from primary, secondary and tertiary infection**. Sera from groups of BALB/c mice, obtained 3–5 weeks after recovery from primary, secondary or tertiary infection by heterotypic or heterosubtypic influenza A viruses, were tested by HeLa-M2 ELISA for M2-specific Ab concentration. Each symbol shows the mean of at least two independent assays, each performed in triplicate or quadruplicate. Cross-bars indicate the geometric mean titer of all groups. B. The same sera were tested for NP-specific Ab titers by ELISA against purified NP.

### Analysis of M2e- and NP-specific Ab responses in humans undergoing a natural IAV infection

Paired serum samples from the acute and convalescent phase of 24 adults presenting with IAV infection and sera from 5 controls were tested for M2e- and NP-specific Ab titers. The assays were performed as for the measurement of these Ab responses in mouse sera except for using i) different serum diluents that helped to reduce the high background binding of human sera (see method section) and ii) a mixture of biotinylated goat-anti-human kappa- and lambda-specific antisera for detection of bound Ab. The M2e-specific Ab titers were expressed in μg/ml in relation to chimeric M2e-specific MAb TRF-3.1. (Note that the difference in M2e sequence at aa position 21 between PR8 (Gly) and most contemporary human IAV strains (Glu) has no known effect on M2e antigenicity). The results showed that M2e-specific Ab titers were very low (or undetectable at 1/20 serum dilution) in acute (GMT = 0.14 μg/ml, n = 24) and control sera (GMT = 0.26 μg/ml, n = 5), i.e. were in the range of the assay sensitivity threshold. The titers increased by ≥ 4-fold (6–120 fold, average 22 fold) in convalescent sera of 11 patients and by <4-fold (0.2 – 3.8-fold, average 1.7) in convalescent sera of 13 patients (Fig 9). The average M2e-specific Ab titer in convalescent sera was 0.56 μg/ml, an increase of 4 fold over the average titer in acute sera. These findings are generally similar to those reported by Black and collaborators [19].

**Figure 9:** **M2e- and NP-specific Ab titers in human sera from the acute and convalescent phase of naturally acquired influenza virus infection**. A and B. Paired sera from the acute and convalescent phase of 24 patients were tested in ELISA against HeLa-M2. M2-specific Ab titers were quantified by comparison to the binding seen with purified M2e-specific mouse-human chimeric Ab TRF-3.1. A. Sera from 11 patients that showed a ≥ 4-fold increase in M2-specific Ab titer between acute and convalescent phase. Each line connects acute and convalescent titers of an individual patient. B. Sera from 13 patients that showed <4-fold increase between acute and convalescent phase. The stipulated horizontal line in panels A and B indicate the threshold of detection. C and D. The same sera were tested in ELISA for NP-specific Ab titers. The titers are expressed relative to one convalescent serum sample with a high NP Ab titer, which was assigned an arbitrary value of 100. C and D show the acute and convalescent NP-specific titers of the same patients shown in A and B, respectively.

The same sera were tested for NP-specific Ab titers. However, as no chimeric NP-specific Ab was available for quantification, these titers were simply expressed relative to an acute serum sample (serum 12B), which displayed a high NP-specific Ab titer and was assigned an arbitrary concentration of 100. On average, the NP-specific titers increased by only 2.5-fold between acute and convalescent phases and only 5 patients showed a ≥ 4-fold increase. In Fig 9, the patients are grouped according to their M2e-specific Ab response into the eleven high (Fig 9C) and thirteen low (Fig 9D) responders. It is evident that the eleven high anti-M2e responders showed on average also a stronger NP-specific response (3.5-fold increase between acute and convalescent phases) than the low responders (1.9-fold increase). Although the M2e- and NP-specific Ab titers in human sera could not be compared directly, the NP-specific titers appeared to be substantially higher than the M2e-specific titers, similar to what was seen in mice after the first and second infection (Fig 8). This was indicated by the fact that the NP- and M2-specific ELISAs showed similar sensitivity (within 3-fold range) for detecting mouse MAbs (Fig 10A), yet detected NP-specific Abs in human sera at ~1000-fold higher dilution than M2-specific Abs (Fig 10B). Thus, human sera appear to contain100-1000-fold higher NP- than M2e-specific Ab titers, e.g. ~0.2 μg/ml anti-M2e and 20–100 μg/ml anti-NP.

**Figure 10:** **Comparison between HeLa-M2 and NP ELISAs**. A. Purified murine MAbs 14C2-S1-4 (anti-M2e, closed circles) and L39-17 (anti-NP, open circles) were tested by ELISA for binding to HeLa-M2 and NP immunosorbents, respectively. Bound MAbs were detected in parallel assays by the same procedure (187-biotin/streptavidin-peroxidase/OPD). Each symbol shows mean OD ± SEM of triplicates. The data are representative of several independently performed assays. B. Five human control sera were tested at various dilutions in ELISA against HeLa-M2, NP and the corresponding control immunosorbents. Bound Abs were detected in parallel assays by the same procedure (biotinylated goat-anti-human cκ,λ/streptavidin-peroxidase/OPD). M2-specific (closed symbols) and NP-specific binding (open symbols) are expressed as Δ ODs. Symbols show means of duplicates. One of two independent assays is shown.

## Discussion

Previous studies indicated poor M2e-specific Ab responses following IAV infection in mice [11,13] and humans [19,20]. It was not clear, however, whether the low responses reflected the inability of the previously used assays to detect the entire repertoire of M2e-specific Abs or whether the M2 presented to the immune system in the context of an infection is poorly immunogenic. To resolve this issue, we developed an ELISA that used M2-transfected HeLa cells as immunosorbent. Assuming that HeLa-cells expressed M2 in the same form as virus-infected host cells, this cellular immunosorbent would be expected to detect all biologically relevant M2-specific Abs. HeLa-M2 cells were shown to express tetrameric M2 (Fig 4A) and were found to be superior to immobilized M2e peptide immunosorbent in detecting M2e-specific Abs induced in mice by repetitive infections (Fig 5C). However, in spite of the improved assay, the HeLa-M2 ELISA reaffirmed that the M2e-specific Ab response was poorly induced by infection. Thus, three consecutive infections were required to raise M2e-specific Ab titers in mice to the level (~50 μg/ml) reached in the NP-specific response after a single infection (Fig 8). In humans, natural infection resulted in a ≥ 4-fold increase in M2e-specific Ab titers in 45% of subjects. However, if induced, the response appeared to be of short duration as M2e-specific Ab titers were very low or undetectable in serum samples obtained from the acute phase of the infection or from controls. Thus, the study confirmed that IAV infection in mouse and human induced a poor M2e-specific Ab response and, more importantly, that humans lacked significant M2e-specific Ab-mediated protection.

Competition binding studies indicated that ~20% of the infection-induced M2e-specific Ab response (in a pooled serum from four mice) that reacted with HeLa-M2 cells, crossreacted with monomeric M2e-peptide. This is most likely the fraction of the total response to native M2e-tetramer that is detected by ELISA using M2e-peptide immunosorbent and is induced by immunization with M2e peptide vaccines that display M2e-peptides in monomeric form.

Although the majority (~80%) of infection-induced M2e-specific Abs did not react with monomeric M2e-peptide, none of the M2e-specific MAbs generated in our laboratory from infection-primed mice reacted exclusively with M2 tetramer (data not shown). This can be explained by the fact that all lymphocyte donor mice were boosted with M2e-MAP prior to fusion – to increase the probability of isolating M2e-specific hybridomas [13] – and initial hybridoma cultures had to be screened for M2e-specific Ab secretion by ELISA against M2e-peptide immunosorbent as the HeLa-M2 cell line was not available at the time. We are currently attempting to isolate M2e tetramer-specific hybridomas from infection-immunized mice without peptide boost and using the HeLa-M2 ELISA for screening. Holsinger and Lamb, 1991 [2] described an MAb that reacted in Western blot with M2 dimer but not M2-monomer and appears to be a member of this dominant M2-polymer-specific Ab group.

The reason for the low M2e-specific Ab response induced by infection remains unknown but the following two factors are likely to contribute. First, the number of naive M2e-specific precursor B cells may be very small and their expansion into a sufficiently large population of M2e-specific Ab-secreting and memory B cells may require several rounds of stimulation. This is consistent with the finding that three consecutive infections in mice were required for induction of M2e-specific Ab titers in the range of 50 μg/ml. It is consistent also with the small size of the antigenic region of M2e. Indeed, the latter may comprise ≤ 15 amino acids [16,20,22], which is in the lower size range of a typical protein epitope recognized by an individual Ab [23]. The small size of the antigenic determinant would be expected to restrict the number of unique combinations of V gene segments that interact strongly with it and thus the number of M2e-reactive B cells in the naive repertoire [22]. Second, antigenic competition by the much more numerous HA- and NA-specific B cells for a limited amount of immunogenic entities may further suppress the M2e-specific Ab response. To participate in a Th-dependent Ab response, antigen-specific B cells must capture the specific antigen with their membrane Ig, internalize and process it and finally display its associated helper T cell determinants to permit cognate interaction with activated helper T cells. As the immunogenic M2e entities may consist predominantly of membrane fragments that contain also associated HA and NA molecules, the much more numerous HA- and NA-specific precursor B cells would be expected to capture and consume most M2, leaving little for stimulation of the few M2e-specific precursor B cells. Antigenic competition by HA-specific precursor B cells has been shown to suppress the NA-specific Ab response both in humans [24] and mice [25]. The phenomenon of antigenic competition was shown to depend on the physical linkage between competing antigens [26, 27] and could be modified by prior immunization against one of the component antigens [27, 28]. The fact that good M2e-specific responses can be induced by immunization with isolated M2e antigen constructs supports a role for antigenic competition in the low M2e-specific Ab response. Still, assuming that most of the adult human serum donors analyzed in this study had experienced several previous IAV infections and in view of the sizeable M2e-specific response seen in mice after three consecutive infections (Fig 8), the low M2e-specific Ab titers in adult human sera are nevertheless surprising. Perhaps induction of substantial and long lasting M2e-specific Ab responses requires massive and consecutive pneumonias as was the case in the experimental mice but may occur only rarely in humans.

## Conclusion

The study showed that on average only ~20% of the M2e-specific Abs, generated in mice by repetitive IAV infections and capable of binding to M2-transfected HeLa cells, reacted also with monomeric M2e peptide. Use of the M2-transfected HeLa cell-based ELISA for determination of M2e-specific Ab titers in human sera convincingly showed that M2e-specific Ab-mediated protection is currently subpoptimal or absent in humans. This provides a strong incentive for the development of an M2e-specific vaccine.

## Methods

### Media and solutions

ISC-CM is Iscove Dulbecco medium (Invitrogen) supplemented with 0.05 mM 2-mercaptoethanol, 0.005 mg/ml transferrin (Sigma), 2 mM L-glutamine (Mediatech-Cellgro) and 0.05 mg/ml gentamicin (Mediatech-Cellgro). ISC-CM was further supplemented with fetal calf serum (FCS, Hyclone Laboratories) or bovine serum albumin (BSA, Sigma) at the indicated concentrations. PFHM-II is protein-free hybridoma medium (Invitrogen). TCRM is phosphate-buffered (pH7.2) potassium/sodium saline supplemented with 2.5 mM EDTA. PBSN is phosphate buffered saline (pH7.2) supplemented with 3 mM NaN3.

### Human and mouse sera

Acute and convalescent sera from humans were obtained during an influenza therapeutic trial in the winter of 1985. Subjects were healthy young adults who presented within 24 hours of onset of clinical influenza with fever (≥ 100°F). Respiratory secretion samples from each subject yielded influenza A (H3N2) virus and paired sera exhibited a significant increase in hemagglutination-inhibiting (HI) antibody between the acute and convalescent sampling. Before submitting the sera for testing for M2e-specific antibody, the HI titers detected in a subset of the sera were confirmed to be unchanged from the original titers. Exempt status (EX2409036-1) for the measurement of Ab titers in blinded paired sera from these studies was granted by the Institutional Review Board of the Wistar Institute,

Naive mouse serum (NMS) was obtained from BALB/c mice. Pooled plasma or serum was obtained from convalescent BALB/c mice (2–5 per group) 21–28 days after primary total respiratory tract infection with A/PR/8/34(H1N1)-Mt.S-Wi (PR8), 10–28 days after secondary and 7–37 days after tertiary infection. The viruses used for consecutive infection shared the same M2e sequence but differed in HA sequence to bypass extant HA-specific immunity [13]. Plasma and serum were also obtained from BALB/c mice that had been inoculated twice by the intranasal or subcutaneous routes with the multiple antigenic peptide vaccine (4)M2e-MAP [13]. An antiserum specific for the intracytoplasmic C terminus of M2 was produced by immunization of mice with the linear peptide T2M2C (AQYIKANSKFIGITEDADDGHFVSIELE, biotech@voicenet.com), which contains on its N-terminus the helper determinant of tetanus toxoid (830–843) [29] and on its C terminus the intracytoplasmic C terminus of M2 of PR8 (underlined in the linear peptide). Ten μg T2M2C, 1 μg cholera toxin (Sigma) and 5 μg immunostimulatory oligodeoxynucleotide 1826 [30], emulsified in 100 μl PBS/50% incomplete Freund adjuvant, were injected twice (3 week interval) into the tail base of five BALB/c mice. Plasma was obtained three weeks after the second injection and pooled. All protocols for animal experiments were approved by the Animal Care and Use Committee of the Wistar Institute.

### Expression of M2 in HeLa Tet-on cells

Full-length M2 cDNA of PR8 was cloned into the BamHI/EcoR V restriction site of pENTR™ TOPO^R ^vector (Invitrogen) and the insert verified by sequence analysis. M2 was subsequently cloned into the BamHI/EcoR V site of the Tet-on response vector pTRE2pur (BD Biosciences) to produce pTRE2pur-M2. A HeLa cell line, stably transfected with the pTet-On regulatory plasmid (BD Biosciences), was maintained in ISC-CM supplemented with 10% Tet system approved FBS (Tet-FBS) (BD Biosciences) and 500 μg/ml G418. For transfection, 10^5 ^Tet-On HeLa cells per ml OptiMem medium were seeded into wells of a 6-well plate and transfected with 4 μg pTRE2pur-M2 using Lipofectamine 2000 (Invitrogen) according to the manufacturer's instructions. After 24 hrs, the cells were resuspended in ISC-CM supplemented with 10% Tet-FBS and 0.5 μg/ml puromycin (BD Biosciences), transferred into 100 × 20 mm petri dishes and maintained in an air/CO_2 _incubator for 2 weeks. Forty well-growing colonies of adherent HeLa cells were harvested by overlaying individual, well separated, colonies with cloning discs (PGC Scientific) soaked with trypsin-versene medium (Sigma) and transferring the disks with adherent cells to individual culture dishes. Replicate samples of individual colonies were seeded into 96-well plates, cultured for 2 days in ISC-CM-10%FCS supplemented with doxycycline (1 μg/ml, BD Biosciences) and then tested by ELISA for expression of M2. The colony with the highest expression level of M2 was selected and expanded in ISC-CM supplemented with 10% Tet-FBS, 0.5 μg/ml puromycin and 500 μg/ml G418. The cell line is reported here as HeLa-M2. A control HeLa cell line stably transfected with empty pTRE2pur was similarly generated and a clone (HeLa-C10) selected based on good growth rate in the presence of the selection marker puromycin.

### ELISA using HeLa-M2 and HeLa-C10 cells

Cells were released from confluent monolayers in T75 flasks by incubation with TCRM and vigorous tapping of the flask. Released cells were suspended at 10^5^/ml in ISC-CM supplemented with 10% FBS and 1 μg/ml doxycycline and dispensed (150 μl/well) into flat bottom 96-well Microtest™ plates (Falcon). After 2 days of incubation at 37°C in air/CO_2_, when the cells had formed closed monolayers, the medium was flicked out and the monolayers were fixed by incubation for 20 min at room temperature with 100 μl 0.05% glutaraldehyde in PBS. The glutaradehyde was then flicked out, the monolayers washed with PBSN and incubated with PBSN-1% BSA (~150 μl/well) for blocking and storage of the plates in the refrigerator.

For ELISA, plates were washed once with PBSN and then sequentially incubated with serum dilutions, biotinylated rat anti-mouse Cκ-specific MAb 187 (ATCC HB58) or a mixture of goat-anti-human Cκ and Cλ-specific antisera (Southern Biotech), streptavidin-peroxidase polymer (Sigma) and o-phenylenediamine dihydrochloride (OPD, Sigma). Sera were diluted in PBSN containing 0.5% gelatin (Sigma) and 0.5% skim milk and tested in triplicate or quadruplicate aliquots at 50 μl/well. Reagents were diluted in PBSN-1% BSA and used at 50 μl/well except for OPD, which was diluted in Sigma Fast buffer and used at 100 μl/well. All washes between sample applications were done with PBSN. The assay was stopped by addition of 50 μl 2 M HCl/well and OD read with the Emax microplate reader (Molecular Devices, Sunnyvale, CA) at 490 and 750 nm and the difference (OD_490–750_) recorded. Assays were performed in parallel on HeLa-M2 and HeLa-C10 immunosorbents, both present in the same assay plate, and the difference in OD_490–750 _between HeLa-M2 and HeLa-C10 computed and recorded as ΔOD. This was necessary because sera, particularly when used at low dilution, displayed substantial and individually distinct levels of background binding as revealed by reaction with HeLa-C10 (background binding was lower when the assay was developed with IgG heavy chain-specific Ab reagents, presumably because Abs of IgM isotype make a dominant contribution to assay background). Assays of murine and human sera were quantified by titration of known concentrations of purified M2e-specific MAb 14C2-S1-4 and the human-mouse chimeric MAb TRF-3.1 (see below), respectively. Data were analyzed with the Softmax software (Molecular Devices).

### Competitive binding assay

The assay was essentially performed as described by Zhang et al., 2006 [22], except for using HeLa cell immunosorbents instead of M2e-peptide immunosorbents. In brief, dilutions of M2e-peptide were mixed with a constant dose of serum or MAb, incubated for 45 min and then transferred to HeLa-M2 and HeLa-C10 immunosorbents. After 45 min incubation, samples were removed and bound Ab detected as in the HeLa ELISA described above. The competing peptide was (2)M2e-MAP, which contains 2 chains of M2e(2–24) attached to a linear Cys-Gly-(Lys-Gly)_4_-Ala backbone [13].

### Trypsin treatment and permeabilization of HeLa immunosorbents

Glutaraldehyde-fixed and BSA-blocked HeLa cell monolayers were extensively washed with warm (37°C) PBS and then incubated for 30 min at 37°C with dilutions of trypsin (2.5%, Gibco) in PBS ranging in 2-fold steps from 1/8 to 1/64. The trypsin was then rinsed off and the immunosorbents were compared by ELISA to untreated HeLa cell monolayers for binding of a saturating dose of M2e-specific MAb or mouse antiserum raised against T2M2C, which contained Abs specific for the intracytoplasmic C-terminus of M2. Glutaraldehyde-fixed and BSA-blocked HeLa-M2 immunosorbents were permeabilized by incubation for 10 min at room temperature with PBSN containing 0.5% NP40. Detergent was then rinsed off and the plates were used in ELISA as described above.

### Analysis of HeLa-M2 by SDS PAGE and Western blot

HeLa-M2 and HeLa-C10 cell monolayers were cultured for 2 days in 6-well cluster plates as described above for preparation of ELISA plates but using 2 ml cell suspension/well. Monolayers were fixed with glutaraldehyde or left unfixed. Monolayers were incubated with 0.5 ml lysis buffer, the lysate was sonicated and electrophoresed under non-reducing conditions in a preformed 10% Tris-Bis polyacrylamide gel (NuPage, Invitrogen) with MES running buffer. The gel was blotted onto a PVDF membrane (Invitrogen). The membrane was blocked with PBSN-1%BSA and stained by sequential incubation with M2e-specific MAb 14C2, biotinylated anti-Cκ MAb 187, streptavidin-peroxidase and diaminobenzidine.

### Expression and purification of recombinant nucleoprotein (rNP)

Full-length NP cDNA of PR8 with 5' EcoRI and 3' NotI restriction sites was inserted into the EcoRI/NotI site of pFast Bac1 HTA vector (Invitrogen), which will encode NP with N-terminal 6xHis tag and intervening TEV recognition site for subsequent enzymatic removal of the His tag. Recombinant baculovirus expressing full-length NP was generated and grown in Sf9 cells. rNP was isolated from infected Sf9 cell lysates using the Y-PER™ 6xHis Column Purification Kit (Pierce) according to the manufacturer's instructions. Purified rNP was quantified by BioRad protein assay and light absorption at 280 nm.

### NP-specific ELISA

Purified rNP (with 6xHis tag) was diluted to 5 μg/ml in 0.02 M NaCl and 25 μl samples were dispensed into 96-well round bottom Serocluster™ polyvinyl plates. The plates were covered with plastic sheets to avoid evaporation, incubated overnight at room temperature and then blocked for 1 hr by incubation with PBSN-1% BSA before use in ELISA. The ELISA procedure was as indicated above for the HeLa ELISA except that 25 μl volumes were used for serum dilutions and reagents and 50 μl for substrate. All samples were tested in parallel against wells coated with rNP and against uncoated BSA-blocked control wells and ΔODs were computed. In the case of human sera, binding activity was expressed relative to serum 12B, which was included as standard in each assay and was assigned an arbitrary NP-specific Ab concentration of 100. In the case of mouse sera, binding activity was expressed relative to purified NP-specific MAb L39-17.

### M2e-peptide-specific ELISA

The multiple antigenic peptide consisting of a Cys-(Gly-Lys)_3_-Ala backbone with two attached M2e(2–24) peptides was used to coat wells of 96-well Microtest™ plates (Falcon) by incubation of 50 μl peptide dilution in 0.02 M NaCl overnight at room temperature. The ELISA was performed as described above for the HeLa-M2 assay.

### Generation of M2e-specific chimeric mouse-human MAb

Cloning of light (L) and heavy (H) chain variable (V) regions of the M2e-specific MAb M2-56, including signal sequences, into the TOPO TA vector (Invitrogen) has been described [22]. V_L _cDNA was amplified with Taq DNA polymerase (Promega) using a forward primer that hybridized to the leader sequence of the V_L _region and contained a Kozak recognition site and EcoR V restriction site 5' of the initiation codon (5' GGGGAT ATCCCACC **ATG**GAGT CACAGA CTCAG 3'; EcoR V site underlined and initiation codon in bold letters) and a reverse primer that hybridized to the Jκ 1 region and contained a Sal I restriction site (5' GTAAGTCGACTTACG**TTT**GATTTCCAGCTTGGTGCC 3'; restriction site underlined, terminal Jκ 1 codon in bold, intervening sequence to provide correct splice site). The PCR product was inserted into the TOPO TA vector and the cloned insert confirmed by EcoR I digestion and sequencing. The TOPO TA vector was then digested with EcoR V and Sal I restriction enzymes (NEB), the V_L _fragment purified by agarose gel electrophoresis and ligated with T4 DNA ligase (NEB) into the EcoR V/Sal I site of the expression vector pAG4622 [31]. The ligation reaction was transformed into E.coli HB101 competent cells (Promega). Ampicillin-resistant colonies were selected on LB agar and amplified in LB/ampicillin medium. Plasmid was extracted with the Qiagen miniprep kit and screened for presence of an insert of correct size by digestion with EcoR V and Sal I and agarose gel electrophoresis. Inserts of selected clones were confirmed by sequence analysis. The resulting expression vector was designated pAG-LK56.1. A similar procedure was followed for cloning of V_H _into the expression vector pAZ6860 [31]. V_H _was amplified with the forward leader sequence primer (5' GGGGATATC CCACC **ATG**GGTTGGAGCTGTATCATC 3'; 5' flanking EcoRV site underlined) and the reverse J_H_3 primer (5' GTAGCTAGC**TGC**AGAGACAGTGACCCAGAGT 3'; Nhe I restriction site underlined and last 3' J_H_3 codon in bold). The PCR product was purified, digested with EcoR V and Nhe I and ligated into the EcoR V/Nhe I site of expression vector pAZ6860. This resulted in the expression vector pAZ-LH56. 10^6 ^X63-Ag8.653 cells [32] in OptiMem were transfected with pAG-LK56.1 and pAZ-LH56 using Fugene 6 (Roche) according to the manufacturer's protocol. The cells were cultured for 2–3 days in OptiMem with 10% FCS and subsequently in medium supplemented with the selection marker zeocin (1 mg/ml). After 2 weeks, residual viable cells were cloned in the same medium by limiting dilution. Medium from well growing clones was tested by ELISA for concentration of M2e-specific Ab, using biotinylated goat-anti-human Cκ-specific antiserum for detection of bound Ab. The clone with highest secretion of M2e-specific MAb (TRF-3.1) was selected.

### Purification of chimeric M2e-specific MAb

TRF-3.1 cells were expanded in ISC-CM supplemented with 5% FCS and Zeocin (1 mg/ml). Cells from dense cultures were pelleted and cultured to exhaustion (~90% cell death) in protein-free PFHM-II medium without zeocin. Cells and debris were pelleted, and chimeric MAb was purified from the medium by adsorption to and elution from a protein G column (Pierce).

## Competing interests

The author(s) declare that they have no competing interests.

## Authors' contributions

JF generated the M2-transfected and control HeLa cell lines and cloned viral NP for expression in the Baculovirus system. MZ generated the chimeric (mouse/human) M2e-specific H and L chain expression vectors and established the chimeric Ab-secreting cell line. KM performed Western blots and ELISAs. DZ participated in the performance of ELISAs. HH expressed NP in the Baculovirus system. WW contributed to the NP expression and editing of the manuscript. RBC collected the human sera and contributed to the editing of the manuscript. WG designed the study, established the cell-based ELISA and was involved in data analyses and preparation of the manuscript.
